This article has been retracted.

# Handgrip Strength-Related Factors Affecting Health Outcomes in Young Adults: Association with Cardiorespiratory Fitness

**DOI:** 10.1155/2021/6645252

**Published:** 2021-04-21

**Authors:** Mingchao Zhou, Fubing Zha, Yuan Chen, Fang Liu, Jing Zhou, Jianjun Long, Wei Luo, Meiling Huang, Shaohua Zhang, Donglan Luo, Weihao Li, Yulong Wang

**Affiliations:** ^1^The First Affiliated Hospital of Shenzhen University, Shenzhen Second People's Hospital, Shenzhen Institutes of Advanced Technology, Chinese Academy of Sciences, Shenzhen, Guangdong, China; ^2^The First Affiliated Hospital of Shenzhen University, Shenzhen Second People's Hospital, Shenzhen, Guangdong, Medical College, Shantou University, Shantou, Guangdong, China; ^3^Shenzhen Dapeng New District Nan'ao People's Hospital, Shenzhen, China

## Abstract

**Objectives:**

Handgrip strength (HS) is a risk factor of all-cause mortality and cardiovascular diseases. However, the influencing factors and mechanisms contributing to this correlation remain unclear. Therefore, we aimed to explore factors related to HS and investigated the mechanism underlying its risk predictive value.

**Methods:**

This was a prospective, cross-sectional study. One hundred forty-five participants were recruited from December 2019 to November 2020. HS was measured using a hydraulic hand dynamometer and adjusted for body mass index (HS_BMI_) and body surface area (HS_BSA_). Body composition was assessed via bioimpedance spectroscopy. Physical fitness was measured using a cardiopulmonary exercise test system. Univariate, multiple linear regression analyses and receiver operator characteristic curve (ROC) were conducted to evaluate the associations between various participant characteristics and HS.

**Results:**

The average participant age was 21.68 ± 2.61 years (42.8% were male). We found positive correlations between HS_BMI_/HS_BSA_ and VO_2max_, VE_max_, Load_max_, and MET_max_ in both sexes (*p* < 0.05). Lean-tissue, protein, total water, and inorganic salt percentages were positively correlated, and fat percentage was negatively correlated with HS_BMI_ in men and with HS_BMI_ and HS_BSA_ in women (*p* < 0.05). Multiple regression revealed that VO_2max_ was independently associated with HS_BSA_ in both sexes (*β* = 0.215, 0.173; 95%confidence interval [CI] = 0.032 − 0.398, 0.026-0.321; *p* = 0.022, 0.022, respectively) and independently associated with HS_BMI_ in women (*β* = 0.016, 95%CI = 0.004 − 0.029, *p* = 0.011). ROC analysis showed that HS_BMI_ and HS_BSA_ can moderately identify normal VO_2max_ in men (area under curve [AUC] = 0.754, 0.769; *p* = 0.002, 0.001, respectively) and marginally identify normal VO_2max_ in women (AUC = 0.643, 0.635; *p* = 0.029, 0.042, respectively).

**Conclusions:**

BMI- and BSA-adjusted HS could serve as indicators of physical health, and HS_BSA_ may moderately reflect cardiorespiratory fitness levels in healthy young adults, particularly in males. Clinical trials registry site and number: China Clinical Trial Center (ChiCTR1900028228).

## 1. Introduction

Handgrip strength (HS) is a simple measurement and a useful indicator of physical strength. HS has been found to be strongly correlated with maximum upper and lower body strength and overall muscle strength [1]. Therefore, HS is commonly used to evaluate sports performance in athletes [2]. In addition, HS is a risk factor for unfavorable health outcomes and is associated with all-cause mortality and cardiovascular diseases (CVD), not only in older individuals but also in young adults [3–5]. Low HS (defined as <26 kg for men and <16 kg for women) is significantly correlated with a high risk of premature mortality, an increased incidence of disability, prolonged length of stay after hospitalization or surgery [6], and high risk of cancer [7]. Therefore, HS measurement can provide abundant information for health assessments [8]. However, the factors or mechanisms underlying the association between HS and health outcomes remain unclear [9].

Previous studies have shown that HS depends on age, sex, body size, socioeconomic status, and physical activity levels [10, 11]; malnutrition and sarcopenia can significantly affect HS [12]. However, these factors are insufficient in explaining the health assessment and risk prediction value of HS. Furthermore, these factors lead to a high heterogeneity of HS between different populations and create difficulty in drawing comparative conclusions among them. Therefore, to more effectively identify HS-related factors affecting health outcomes, HS adjusted for body mass index and body surface area (HS_BMI_/HS_BSA_) has been used to reduce the influence of heterogeneity on the results [13].

VO_2max_, a representation of cardiorespiratory fitness (CRF), is closely correlated to physical health. Low VO_2max_ is recognized as a strong and independent risk factor for all-cause mortality, CVD [14], diabetes mellitus [15], and neoplasia [16] in healthy adults, and accordingly, VO_2max_ was consistent with HS affecting health outcomes in healthy population [17, 18]. A recent study indicated a strong association between HS and VO_2max_ in paraplegic men [12]. Therefore, we speculate that HS and CRF may be correlated with each other, thereby interactively affecting the health outcomes in the general population. The aforementioned factors may influence HS and contribute to the risk predictive value of HS. The aim of this study was to explore the potential indicators associated with HS, especially the possible interrelationships between HS and CRF.

## 2. Materials and Methods

### 2.1. Study Design

This was a prospective, cross-sectional study. This study is part of the “Study for the application value of grip strength on the unaffected side in patients with stroke”, which involves two steps. The first step is to explore the correlation between HS and CRF in healthy young adults, the aim of the current study. The next step is to test whether the association between grip strength and cardiorespiratory fitness persists in stroke patients, which will be undertaken in the future. Our overall goal is to extrapolate the associations found in healthy young adults to stroke patients and to provide a useful predictive tool for stroke patients who have difficulty undertaking cardiopulmonary exercise tests. In the current study, the data were obtained from the rehabilitation center of Shenzhen Second People's Hospital and Shenzhen Dapeng New District Nan'ao People's Hospital, Shenzhen City, China. This study conforms to the standards of the Declaration of Helsinki, was approved by the Ethics Committee of Shenzhen Second People's Hospital (KS20191119005), and was registered at the China Clinical Trial Center (ChiCTR1900028228).

### 2.2. Participants

Study participants were recruited using a convenience sample of young adult interns in the hospital. Based on the sample size calculation method for a multiple regression study (https://www.danielsoper.com), a minimum sample size of 70 participants of each sex was needed to achieve 90% power and to detect an effect size (Cohen's *f*^2^) of 0.26 attributable to 5 independent variables using an *F*-Test (multiple regression analysis) with a significance level (alpha) of 0.05. Combined with a 10% shedding rate, 154 subjects were needed for this study. The participants were recruited from December 2019 to November 2020 based on the following inclusion and exclusion criteria. The inclusion criterion was healthy young adults (aged 18–24 years) with a stable physical condition. The exclusion criteria were (1) congenital heart disease, (2) history of cardiac arrest, (3) neurological or muscular disorders, (4) fever or infection, and (5) allergy to electrode pads. Before data collection, participants were informed of the objectives and methodology of the study, and written informed consent was obtained. Tea or coffee was prohibited for at least 3 h before the tests. Tests were performed in an evaluation room with a temperature of 22–25°C. Except for scientific purposes, personal information and experimental data were kept strictly confidential.

### 2.3. Variables

Data for the following parameters were recorded within 72 hours after admission (baseline): (1) demographic factors, such as sex and age (years); (2) anthropometric factors, such as height (m), weight (kg), body mass index (BMI, kg/m^2^), body surface area (BSA), and resting heart rate (HR_rest_, bpm); (3) body composition, including lean-tissue percentage (%), fat percentage (%), protein percentage (%), total water percentage (%), and inorganic salt percentage (%); (4) physical fitness, including AT (ml/kg·min), VO_2max_ (ml/kg·min), HR_rest_ (rpm), HR_AT_ (rpm), HR_max_ (rpm), RER_max_, VE_max_ (ml/min), Load_max_ (W), Psys_max_ (mmHg), Pdia_max_ (mmHg), MET_max_, *ΔV*O_2_/*Δ*Load, ventilatory equivalent for carbon dioxide (VE/VCO_2_), and oxygen uptake efficiency slope (OUES); and (5) living habits, such as smoking status (current smoker or nonsmoker) and exercise habits (sedentary, exercise 1–2 times a week, exercise ≥3 times a week). BMI was calculated as body weight/height in meters squared (kg/m^2^). BSA was calculated using Mosteller formula [$\text{BSA}\left({\text{m}}^{2}\right)=\sqrt{\text{heigth}\left(\text{cm}\right)\times \text{weigth}\left(\text{kg}\right)/3600}$] [19]. HR_rest_ was calculated as the average heart rate during 10 min of quiet sitting. Body compositions were measured using a body bioimpedance spectroscopy (X-one; Youjiu, Shanghai, China). Physical fitness was measured via a cardiopulmonary exercise test (CPET) evaluation system (MasterScreen; Ergoline, Germany).

### 2.4. Handgrip Strength Test

HS was measured using a hydraulic hand dynamometer (Jamar, 1516801, Patterson Medical Ltd, UK). Based on previous authoritative research [20], the standard measurement process for HS is described as follows. The participants were seated upright with their elbow flexed at a 90°angle, with the forearm facing forward and resting on a table or an armrest. After taking the hand dynamometer, the participants were asked to complete a maximal handgrip effort two or three times on each side, expressed in absolute units (kg). Each measurement was completed at least 1 min apart to allow full muscle strength recovery. The average value of each measurement was recorded as the normal HS of one side (HS_left_ and HS_right_), and the mean of the right- and left-side values was recorded as the average HS (HS_average_). HS is partly associated with body size [21]; therefore, to prevent this association from influencing the results, we adjusted the HS_average_ for BMI and BSA and created two new indicators, HS_BMI_ and HS_BSA_, respectively.

### 2.5. Cardiopulmonary Exercise Test

In accordance with the “Clinician's Guide to Cardiopulmonary Exercise Testing in Adults: A Scientific Statement from the American Heart Association” [22], the graded, symptom-limited maximal cardiopulmonary exercise test (CPET) was used to measure CRF via an incremental cycle ergometer (MasterScreen; Ergoline, Germany). CRF is reflected by maximum level of oxygen consumption (VO_2max_) [5]. Gas exchange measurements were conducted through breath-by-breath analysis using the Jaeger Carefusion system (V-706575; Jaeger, Germany). Heart rate was monitored throughout testing via a 12-lead electrocardiogram (ECG). Before testing, participants were instructed to rest for 10 min. Subsequently, participants were instructed to sit on the cycle ergometer and were fitted with a face mask, ECG, and sphygmomanometer. Then, they were instructed to complete the following measurement processes: (1) 3 min phase of seated rest, (2) 3 min phase of cycling without resistance, (3) 8–12 min phase of cycling with an increasing work rate from zero to their individual peak power (the cycling work rate was increased by one-tenth of the predicted maximum power calculated by the machine according to age, sex, height, and weight), (4) 3 min recovery period at a constant power of 20 W, and (5) 3 min phase of seated recovery. During the entire cycling period, the participants were asked to cycle at a constant speed of 60 rpm.

Oxygen uptake at maximum load was recorded for each participant as VO_2max_ (ml/kg·min). According to previous studies [23], in male young adults (15 to 30 years old), VO_2max_ < 30 ml/kg · min is defined as abnormal, and VO_2max_ ≥ 30 ml/kg · min is normal. In female young adults, VO_2max_ < 25 ml/kg · min is regarded as abnormal, and VO_2max_ ≥ 25 ml/kg · min is normal. The anaerobic threshold (AT) was determined by the V-slope and ventilatory equivalents methods [5]. AT is the departure point of VO_2_ from a line of identity drawn through a plot of VCO_2_ versus VO_2_ in the V-slope method, as well as the point at which a systematic increase in the ventilatory equivalent for oxygen (VE/VO_2_) occurs without an increase in the VE/VCO_2_ in the ventilatory equivalent method [24]. The results of the V-slope method and ventilatory equivalents method were cross-referenced to make the final determination of AT. OUES is calculated by the equation VO2 = *a* log_10_VE + *b* (*a* as OUES), which can reflect the linear relationship between logarithmically transformed VE and VO_2_ [25]. During the testing period, if dizziness, chest tightness, or syncope occurred, the test was stopped immediately, the participant was transferred to a supine position, and a rescue process was initiated, if necessary. Tests were conducted by two experienced physicians who underwent standardized training.

### 2.6. Statistical Analyses

Continuous variables with a normal distribution are expressed as mean ± standard deviation (SD). Categorical variables are expressed as frequency or percentage. The sample size was calculated based on the recorded numbers and reference to an earlier study [26]. Participants with missing important data (e.g., HS, VO_2max_) were excluded from the final analysis. Secondary indicators that were partially missing were filled in with a mean value. The correlation between HS_BMI_ and HS_BSA_ and other characteristics were analyzed by Pearson or Spearman analysis. Multivariate linear regression analysis was conducted to explore factors independently correlated with HS_BMI_ and HS_BSA_. To avoid potential multicollinearity, once a variable had been used to adjust for other variables, it was not included as a covariate in the multivariate linear regression analysis. The receiver operating characteristic curve (ROC) was used to investigate the relationship between sensitivity and specificity. The optimal cutoff scores of HS_BMI_ and HS_BSA_ were determined as the score with the highest sum of sensitivity and specificity. The area under the curve (AUC) was calculated to identify the discrimination potential of HS_BMI_ and HS_BSA_ cutoff score in normal VO_2max_. Because male and female young adults differ substantially in terms of muscular fitness and CRF, statistical analyses were performed separately to analyze the different variables related to HS_BMI_/HS_BSA_ in the two sexes. Analyses were performed using SPSS version 21.0 (Armonk, NY: IBM Corp.). Figures were processed using GraphPad Prism version 6.01 (San Diego, USA). Two-sided *p* values < 0.05 were considered statistically significant.

## 3. Results

### 3.1. Characteristics of Selected Participants

The study flowchart is shown in Figure 1. In the present study, 156 healthy young adults were screened for potential eligibility. After excluding subjects with fever (*n* = 2), arrhythmia (*n* = 1), refusal (*n* = 3), and missing important data (*n* = 5), 145 (62 male, 83 female) healthy, Chinese young adults (average age 21.68 ± 2.61 years) were included for the final data analysis. Basic and anthropometric-related characteristics of the included participants are summarized in Table 1. Results showed that HS-related factors (HS_left_, HS_right_, and HS_average_), body composition-related factors (lean-tissue percentage, protein percentage, total water percentage, and inorganic salt percentage) and CRF-related factors (VO_2max_, VE_max_, Load_max_, and MET_max_) in males were much higher than those in females (*p* < 0.05). Conversely, the fat percentage and resting heart rate in males were much lower than those in females (*p* < 0.05), indicating that muscular fitness, body composition, and CRF were much different between male and female young adults in this study. Therefore, it was necessary to analyze male and female participant data separately.

### 3.2. Univariate Correlations among Characteristics with HS_BMI_ and HS_BSA_

The results of the correlation analysis are presented in Table 2. In young male adults, body composition including lean-tissue percentage, fat percentage, protein percentage, total water percentage, inorganic salt percentage, and CRF-related factors (VO_2max_, VE_max_, Load_max_, and MET_max_) were all significantly correlated with HS_BMI_ and HS_BSA_ (*p* < 0.05). In young female adults, body composition, including lean-tissue percentage, fat percentage, protein percentage, total water percentage, and inorganic salt percentage, were all significantly correlated with HS_BMI_ (*p* < 0.05). Furthermore, CRF-related factors (VO_2max_, VE_max_, Load_max_, and MET_max_) were all significantly correlated with HS_BMI_ and HS_BSA_ (*p* < 0.05). These results reflected that HS_BMI_ and HS_BSA_ were associated with various health-related indicators and had the potential to reflect overall health conditions.

### 3.3. Multiple Regression Analysis among Characteristics with HS_BMI_ and HS_BSA_

Multivariate linear regression analysis was performed to analyze the independent association among HS_BMI_, HS_BSA_ with anthropometric variables, and CRF-related variables. Based on the results of the univariate correlation analysis, having excluded factors of collinearity, the dominant factors correlated with HS_BMI_ and HS_BSA_ were selected into the multivariate linear regression. As shown in Table 3, in males, fat percentage was negatively associated with HS_BMI_ independently (*β* = −2.712, 95%CI = −5.349–−0.075, *p* = 0.044), and VO_2max_ was positively associated with HS_BSA_ independently (*β* = 0.215, 95%CI = 0.032 − 0.398, *p* = 0.022). In females, VO_2max_ was positively associated with both HS_BMI_ and HS_BSA_ independently (*β* = 0.016, 0.173; 95%CI = 0.004 − 0.029, 0.026-0.321; *p* = 0.011, 0.022).

### 3.4. Linear Regression Analysis of HS_BMI_ and HS_BSA_

The results of the linear regression analysis are presented in Figure 2. In male participants, HS_BMI_ explained 20.7% of the variance of VO_2max_ (*R*^2^ = 0.207, *p* < 0.001), and HS_BSA_ explained 21.4% of the variance of VO_2max_ (*R*^2^ = 0.214, *p* < 0.001). While in female participants, HS_BMI_ explained 5.9% of the variance of VO_2max_ (*R*^2^ = 0.059, *p* = 0.027), and HS_BSA_ explained 7.1% of the variance of VO_2max_ (*R*^2^ = 0.071, *p* = 0.015).

### 3.5. Receiver Operating Characteristic (ROC) Analysis of HS_BMI_ and HS_BSA_

The results of ROC analysis are presented in Figure 3. In male participants, the optimal cutoffs in HS_BMI_ and HS_BSA_ used to distinguish a normal level of VO_2max_ were 2.17 and 33.83 (sensitivity = 40%, 80%, respectively; specificity = 100%, 70.6%, respectively), with an area under the curve (AUC) of 0.754 and 0.769 (*p* = 0.002, 0.001, respectively). In female participants, the optimal cutoffs in HS_BMI_ and HS_BSA_ used to distinguish a normal level of VO_2max_ were 1.17 and 15.86 (sensitivity = 66.0%, 56.6%; specificity = 63.3%, 70.0%, respectively), with an AUC of 0.643 and 0.635 (*p* = 0.029, 0.042, respectively).

## 4. Discussion

In this study, we explored factors associated with HS to identify potential mechanisms underlying health outcomes in healthy young adults. Our results indicated that several types of health-related factors, including body composition, physical fitness, and CRF, were correlated with HS_BMI_ and HS_BSA_. Multivariate regression analysis revealed that VO_2max_ was independently associated with HS_BSA_ in both male and female young adults. These findings confirm HS as an indicator of physical health and reveal the possible mechanism underlying the risk predictive value of HS.

HS is affected by many demographic factors, such as age, sex, and BMI. The highest HS scores typically occur between the ages of 24 and 39 years. During normal aging, HS will decrease due to changes in anabolic resistance and reduced physical activity participation [27]. Riviati et al. found that being older than 75 years was associated with lower HS [12]. Besides, Khalid et al. revealed that BMI was positively correlated with HS [28]. Therefore, to eliminate the age-related effects, a population with a narrow age range was selected for the current study. And HS was adjusted for BMI and BSA to allow comparative analyses according to different body weights or sizes.

Anthropometric indicators also influence HS. In the current study, lean-tissue percentage, protein percentage, total water percentage, and inorganic salt percentage were positively correlated with HS_BMI_ and HS_BSA_. Our findings are consistent with an earlier study, in which HS was positively correlated with lean tissue mass, lean tissue index, and serum albumin level in hemodialysis patients [29]. The possible mechanism for these associations may be that muscle mass forms the basis of strength, and protein, inorganic salt, and water establish the nutrition required for HS [30]. Conversely, it is known that a high body fat percentage is strongly correlated with cardiovascular and cerebrovascular diseases because of lipid-induced atherosclerosis [31]. In this study, body fat percentage was negatively associated with HS_BMI_ and HS_BSA_; therefore, these associations may explain why a low level of HS is correlated with high cardiovascular risk [32]. Furthermore, in our study, we found, through multiple regression analysis, that almost all the associations between HS and body composition were covered by VO_2max_, indicating that the relationship between HS and CRF was more stable than that between HS and other factors.

Previous studies have indicated a close association between HS and cardiovascular health and cardiac structure and function [33–35]. Beyer et al. found that a higher HS was associated with a higher left ventricular end-diastolic volume, higher left ventricular stroke volume, lower left ventricular mass, and lower left ventricular mass-to-volume ratio in UK adults [36]. Further, other studies have found that a lower HS may contribute to heart failure with a preserved ejection fraction through the pathways of the activation of systemic inflammation [37] and insulin resistance [38, 39]. Moreover, Zhang et al. reported that HS demonstrated a strong correlation with the six-minute walk test distance in older participants (*R* = 0.549, *p* ≤ 0.001) [26], which is consistent with our findings. These relationships help establish the foundation of the association between HS and CRF. Based on these findings, it may be promising to develop predictive models of VO_2max_ with nonexercise factors in frail populations in the future [40, 41].

The mechanism underlying the association between HS and CRF remains unclear. As reported in the literature, pyruvate dehydrogenase (PDH) might be one of the links. Love et al. found that PDH phosphatase activity is associated with muscle aerobic capacity [42]. Muscle PDH phosphatase was found to be decreased in patients with low HS [43]. Additionally, aerobic training can increase PDH activity and improve maximal capacity to utilize carbohydrates in human skeletal muscle [44].

An interesting finding of this study was that the association between HS_BMI_/HS_BSA_ and CRF was strong in young male adults but weak in young female adults. This may be because HS is strongly influenced by the heritability of sexually dimorphic traits [45], ranging between 50% and 65% for adult males, which is considerably lower for women (30%) [46]. Another reason may lie in the androgenic influences in the development of physical strength. Isen et al. found that, compared with girls, boys experience much more additive genetic effects of changes in HS during the period of adolescence (80% vs. 28%) [44]. Similarly, HS levels in men were much higher than that in women in our study. Meanwhile, because VO_2max_ level is the result of the combined effect of muscle strength and heart and lung function during extreme exercise, and because HS is strongly associated with overall muscle strength [1], the dominance of HS in men may result in a more significant relationship between HS and CRF than in women. These findings suggested that HS may be a good indicator of CRF in men but not necessarily in women.

The clinical significance of this study lies in the following. First, the close relationship between BMI- and BSA-adjusted HS and VO_2max_ may partly explain why HS is a risk factor of all-cause mortality and cardiovascular diseases. Second, the results provide evidence to support muscle strength training as a means to improve CRF. Third, HS, as a simple evaluation index, can moderately reflect the level of CRF and accordingly may act as a potential predictor of CRF levels in frail populations or communities where cardiopulmonary exercise testing is not possible.

There are some limitations to the present study. First, our research subjects were young healthy Chinese adults within a narrow age range limiting generalization to other populations. In future studies, subjects from different age groups should be included. Moreover, we excluded participants with congenital heart disease, a history of cardiac arrest, and muscular disorders. Therefore, the findings of this study cannot be generalized to people with these conditions. Finally, our sample size was small. Future studies with larger sample sizes are necessary to ensure generalizability of the findings.

## 5. Conclusions

Our results showed that HS_BMI_ and HS_BSA_ were correlated with various health-related indicators, including body composition factors (e.g., lean-tissue, protein, total water, and inorganic salt percentage) and CRF factors (e.g., VO_2max_, VE_max_, Load_max_, and MET_max_). HS_BSA_ was independently associated with VO_2max_ levels, especially in males. These associations may partly explain why HS is correlated with health risks. Therefore, we suggest that HS_BMI_ and HS_BSA_ could serve as indicators of physical health, and HS_BSA_ could be used to partially reflect CRF levels in healthy young adults. Larger studies are required to strengthen our conclusions and explore the application value of HS in varied populations.

## Figures and Tables

**Figure 1:** Study flowchart.

**Figure 2:** Linear regression between HS_BMI_ and HS_BSA_ with VO_2max_ in male and female young adults. (a) Linear regression between HS_BMI_ and VO_2max_ in male participants (*R*^2^ = 0.207, *p* < 0.001). (b) Linear regression between HS_BSA_ and VO_2max_ in male participants (*R*^2^ = 0.214, *p* < 0.001). (c) Linear regression between HS_BMI_ and VO_2max_ in female participants (*R*^2^ = 0.059, *p* = 0.027). (d) Linear regression between HS_BSA_ and VO_2max_ in female participants (*R*^2^ = 0.071, *p* = 0.015). BMI: body mass index; BSA: body surface area; HS_BMI_: HS_average_ adjusted for BMI; HS_BSA_: HS_average_ adjusted for BSA; VO_2max_: maximum oxygen uptake.

**Figure 3:** ROC analysis of the associations among HS_BMI_ and HS_BSA_ with VO_2max_ in male and female young adults. (a) The ROC curve between VO_2max_ and HS_BMI_ and HS_BSA_ in male participants. (b) The ROC curve between VO_2max_ and HS_BMI_ and HS_BSA_ in female participants. BMI: body mass index; BSA: body surface area; HS_BMI_: HS_average_ adjusted for BMI; HS_BSA_: HS_average_ adjusted for BSA; VO_2max_: maximum oxygen uptake; AUC: area under curve.

**Table 1:** Characteristics of the study participants.

Characteristics	Male (*n* = 62)	Female (*n* = 83)	*p* value
Demography	Mean ± SD	Mean ± SD	
Age (years)	22.01 ± 3.06	21.44 ± 2.21	0.217
Height (cm)	172.37 ± 6.95	161.05 ± 5.52	≤0.001
Weight (kg)	64.87 ± 10.06	52.64 ± 7.51	≤0.001
BMI (kg/m^2^)	21.80 ± 3.05	20.20 ± 2.31	≤0.001
BSA (m^2^)	1.76 ± 0.15	1.53 ± 0.12	≤0.001
HS			
HS_left_ (kg)	42.56 ± 7.02	24.29 ± 4.53	≤0.001
HS_right_ (kg)	42.81 ± 7.72	24.78 ± 4.95	≤0.001
HS_average_ (kg)	42.69 ± 6.98	24.54 ± 4.39	≤0.001
HS_BMI_	1.99 ± 0.41	1.23 ± 0.24	≤0.001
HS_BSA_	24.38 ± 4.17	16.05 ± 2.71	≤0.001
Anthropometry			
Lean-tissue percentage (%)	0.74 ± 0.04	0.68 ± 0.03	≤0.001
Fat percentage (%)	0.22 ± 0.06	0.28 ± 0.03	≤0.001
Protein percentage (%)	0.17 ± 0.01	0.16 ± 0.01	≤0.001
Total water percentage (%)	0.57 ± 0.03	0.52 ± 0.03	≤0.001
Inorganic salt percentage (%)	0.05 ± 0.01	0.05 ± 0.01	≤0.001
Cardiorespiratory fitness			
AT (ml/kg·min)	18.78 ± 4.72	15.23 ± 3.43	≤0.001
VO_2max_ (ml/kg·min)	33.38 ± 6.28	26.49 ± 4.25	≤0.001
HR_rest_ (rpm)	80.76 ± 14.60	88.66 ± 12.84	≤0.001
HR_AT_ (rpm)	123.97 ± 15.57	126.22 ± 15.66	0.392
HR_max_ (rpm)	174.10 ± 17.49	173.57 ± 12.89	0.841
RER_max_	1.25 ± 0.12	1.23 ± 0.17	0.317
VE_max_ (ml/min)	75.63 ± 19.55	51.77 ± 11.56	≤0.001
Load_max_ (W)	179.79 ± 33.28	109.89 ± 16.83	≤0.001
Psys_max_ (mmHg)	167.24 ± 26.50	138.94 ± 17.40	≤0.001
Pdia_max_ (mmHg)	74.85 ± 13.28	69.00 ± 11.90	0.007
MET_max_	9.54 ± 1.79	7.57 ± 1.22	≤0.001
*Δ*VO_2_/*Δ*Load	10.31 ± 1.26	10.24 ± 1.23	0.741
VE/VCO_2_	24.17 ± 3.38	27.27 ± 3.16	≤0.001
OUES	2224.47 ± 475.02	1647.63 ± 1437.16	≤0.001
Smoking^∗^*N* (%)	49 (79.0)	79 (95.2)	0.003
Exercise habits^∗^*N* (%)			≤0.001
Sedentary	29 (46.8)	65 (78.3)	
1–2 times a week	20 (32.3)	17 (20.5)	
≥3 times a week	13 (21.0)	1 (1.2)	

SD: standard deviation; BMI: body mass index; BSA: body surface area; HS_left_: handgrip strength of the left hand; HS_right_: handgrip strength of the right hand; HS_max_: maximum handgrip strength of the two hands; HS_average_: average handgrip strength of both hands; HS_BMI_: HS_average_ adjusted for BMI; HS_BSA_: HS_average_ adjusted for BSA; AT: anaerobic threshold; VO_2max_: max oxygen uptake; HR_rest_: resting heart rate; HR_AT_: heart rate at anaerobic threshold; HR_max_: max heart rate; Load_max_: max work load; RER_max_: respiratory exchange ratio at max work load; VE_max_: minute ventilation at max work load; Psys_max_: systolic pressure at max work load; Pdia_max_: diastolic pressure at max workload; MET_max_: metabolic equivalent at max work load; *Δ*VO_2_/*Δ*Load: oxygen required at each load; VE/VCO_2_: the minute ventilation/carbon dioxide production slope; OUES: oxygen uptake efficiency slope. Values are shown as mean ± SD or as number (%).

**Table 2:** Univariate correlations between subject characteristics and HS_BMI_ and HS_BSA_.

Characteristics	Male (*n* = 62)		Female (*n* = 83)	
	HS_BMI_	HS_BSA_	HS_BMI_	HS_BSA_
	*r* (*p* value)	*r* (*p* value)	*r* (*p* value)	*r* (*p* value)
Age (years)	-0.021 (0.869)	-0.004 (0.974)	0.001 (0.998)	-0.003 (0.978)
Anthropometry				
Lean tissue percentage (%)	0.568 (≤0.001)	0.459 (≤0.001)	0.286 (0.010)	0.194 (0.083)
Fat percentage (%)	-0.576 (≤0.001)	-0.441 (0.002)	-0.286 (0.010)	-0.171 (0.127)
Protein percentage (%)	0.57 (≤0.001)	0.467 (≤0.001)	0.285 (0.010)	0.190 (0.089)
Total water percentage (%)	0.577 (≤0.001)	0.468 (≤0.001)	0.287 (0.009)	0.204 (0.068)
Inorganic salt percentage (%)	0.494 (≤0.001)	0.383 (0.008)	0.241 (0.030)	0.138 (0.220)
Cardiorespiratory fitness				
AT (ml/kg·min)	0.158 (0.219)	0.188 (0.143)	0.062 (0.579)	0.123 (0.269)
VO_2max_ (ml/kg·min)	0.454 (≤0.001)	0.463 (≤0.001)	0.242 (0.028)	0.267 (0.015)
HR_rest_ (rpm)	-0.282 (0.026)	-0.332 (0.008)	-0.055 (0.619)	-0.024 (0.826)
HR_AT_ (rpm)	-0.232 (0.070)	-0.250 (0.050)	0.021 (0.850)	0.050 (0.657)
HR_max_ (rpm)	0.092 (0.478)	0.092 (0.475)	0.188 (0.089)	0.208 (0.059)
RER_max_	0.181 (0.160)	0.139 (0.280)	0.125 (0.259)	0.081 (0.465)
VE_max_ (ml/min)	0.381 (0.002)	0.344 (0.006)	0.236 (0.032)	0.254 (0.020)
Load_max_ (W)	0.342 (0.007)	0.340 (0.007)	0.201 (0.069)	0.191 (0.083)
Psys_max_ (mmHg)	-0.068 (0.602)	-0.015 (0.908)	-0.254 (0.020)	-0.182 (0.100)
Pdia_max_ (mmHg)	0.049 (0.703)	-0.005 (0.969)	0.100 (0.369)	0.131 (0.237)
MET_max_	0.452 (≤0.001)	0.462 (≤0.001)	0.242 (0.027)	0.265 (0.016)
*Δ*VO_2_/*Δ*Load	-0.147 (0.256)	-0.107 (0.406)	-0.049 (0.657)	-0.008 (0.943)
VE/VCO_2_	0.243 (0.057)	0.147 (0.254)	0.175 (0.114)	0.205 (0.063)
OUES	0.005 (0.970)	0.081 (0.531)	0.079 (0.479)	-0.033 (0.769)
Life habit				
Smoking	0.081 (0.532)	-0.006 (0.966)	0.061 (0.584)	0.120 (0.281)
Exercise habits	-0.105 (0.418)	-0.101 (0.435)	0.125 (0.260)	0.166 (0.134)

SD: standard deviation; BMI: body mass index; BSA: body surface area; HS_left_: handgrip strength of the left hand; HS_right_: handgrip strength of the right hand; HS_max_: maximum handgrip strength of the two hands; HS_average_: average handgrip strength of both hands; HS_BMI_: HS_average_ adjusted for BMI; HS_BSA_: HS_average_ adjusted for BSA; AT: anaerobic threshold; VO_2max_: max oxygen uptake; HR_rest_: resting heart rate; HR_AT_: heart rate at anaerobic threshold; HR_max_: max heart rate; Load_max_: max work load; RER_max_: respiratory exchange ratio at max work load; VE_max_: minute ventilation at max work load; Psys_max_: systolic pressure at max work load; Pdia_max_: diastolic pressure at max work load; MET_max_: metabolic equivalent at max work load; *Δ*VO_2_/*Δ*Load: oxygen required at each load; VE/VCO_2_: the minute ventilation/carbon dioxide production slope; OUES: oxygen uptake efficiency slope. ^∗^*r* for categorical variables: Spearman's correlation coefficient; *r* for continuous variables: Pearson's correlation coefficient.

**Table 3:** Multivariate regression analysis on the associations between subject characteristics and HS_BMI_ and HS_BSA_.

Models	HS_BMI_		HS_BSA_	
	*β* (95% CI)	*p* value	*β* (95% CI)	*p* value
Male (*n* = 62)				
Age (years)	-0.005 (-0.018, 0.027)	0.686	-0.059 (0.419, 0.300)	0.740
VO2max (ml/kg·min)	0.016 (-0.002, 0.033)	0.073	0.215 (0.032, 0.398)	0.022
Lean-tissue percentage (%)	30.457 (-0.121, 70.035)	0.056	140.276 (-270.907, 560.459)	0.498
Fat percentage (%)	-20.712 (-50.349, -0.075)	0.044	-90.401 (-400.043, 210.240)	0.539
BMI (kg/m^2^)	—	—	-0.200 (-0.767, 0.367)	0.480
BSA (m^2^)	0.514 (-0.315, 10.342)	0.200	—	—
Female (*n* = 83)				
Age (years)	0.005 (-0.018, 0.027)	0.686	0.046 (-0.221, 0.312)	0.734
VO2max (ml/kg·min)	0.016 (0.004, 0.029)	0.011	0.173 (0.026, 0.321)	0.022
Lean-tissue percentage (%)	10.452 (-0.402, 30.306)	0.123	80.568 (-140.291, 310.427)	0.458
Fat percentage (%)	-10.805 (-30.712, 0.101)	0.063	-80.210 (-320.635, 160.216)	0.505
BMI (kg/m^2^)	—	—	0.046 (-0.328, 0.420)	0.807
BSA (m^2^)	0.475 (-0.044, 0.993)	0.072	—	—

*β*: effect size; CI: confidence interval; HS: maximum handgrip strength of the two hands; BMI: body mass index; BSA: body surface area; HS_BMI_: HS_average_ adjusted for BMI; HS_BSA_: HS_average_ adjusted for BSA; VO_2max_: maximum oxygen uptake.

## Data Availability

All data used during the study are available from the corresponding author by request.

## Supplementary Materials

Supplementary Materials Supplementary Material 1: STROBE checklist for cross-sectional study. Supplementary Material 2: ethical approval document.
